The article "Nonalcoholic Fatty Liver Hepatocyte-Derived lncRNA MALAT1 Aggravates Pancreatic Cell Inflammation via the Inhibition of Autophagy by Upregulating YAP" was retracted in 2023. Reasons: unreliable results or conclusions; concerns about the data; concerns about the results or conclusions; concerns about the peer review.

# Nonalcoholic Fatty Liver Hepatocyte-Derived lncRNA MALAT1 Aggravates Pancreatic Cell Inflammation via the Inhibition of Autophagy by Upregulating YAP

**DOI:** 10.1155/2022/2930960

**Published:** 2022-08-31

**Authors:** Di Liu, Weijie Yao, Kejun Liu, Genwang Wang, Bendong Chen, Zuozheng Wang, Shaozhang Hou

**Affiliations:** ^1^Department of Hepatobiliary Surgery, General Hospital of Ningxia Medical University, Yinchuan 750004, China; ^2^School of Basic Medical Sciences, Ningxia Medical University, Yinchuan 750004, China

## Abstract

**Background:**

Acute pancreatitis (AP) is one of the most common gastrointestinal disorders, which causes death with a high mortality rate of about 30%. The study aims to identify whether the nonalcoholic fatty liver disease (NAFLD)-derived lncRNA MALAT1 participates in the inflammation of pancreatic cell and its potential mechanism.

**Methods:**

The NAFLD cell model was constructed by treating HepG2 cells with FFA. The *in vitro* model of acute pancreatitis (AP) was established by the administration of caerulein on AR42J cells. MALAT1 and si-MALAT1 were transfected into pancreatic cells, and then exosomes were collected from the NAFLD cell model and then were cocultured with AR42J cells. Transmission electron microscopy was used to observe the morphology of exosomes. Oil Red O staining was applied to reveal the lipid deposition. The triglyceride, IL-6, and TNF-*α* levels were detected using ELISA. The MALAT1 level in exosomes was detected by qRT-PCR. The CD9, CD63, CD81, and CYP2E1, LC3II, and LC3I levels were detected by western blot.

**Results:**

MALAT1 was upregulated in NAFLD-derived exosomes and increased the levels of IL-6 and TNF-*α* in pancreatic cells. NAFLD-derived exosomes inhibited YAP phosphorylation, decreased the levels of IL-6 and TNF-*α*, and reduced the ratio of LC3II/LC3I protein in pancreatic cells. Silencing MALAT1 significantly returned the inhibitory effect of NAFLD on hippo-YAP pathway. YAP1 signal transduction inhibitor CA3 reversed the decrease of LC3II/LC3I expression and the increase of IL-6 and TNF-*α* levels induced by MALAT1 in the AP cell model.

**Conclusions:**

NAFLD-derived MALAT1 exacerbates pancreatic cell inflammation via inhibiting autophagy by upregulating YAP.

## 1. Introduction

Acute pancreatitis (AP) is able to cause death with high mortality rate of about 30%, which is one of the most common gastrointestinal disorders [1–3]. Pancreatic necrosis/apoptosis and systemic inflammation are the characteristics of AP [4]. Over the centuries, several studies have been conducted on the etiology and pathogenesis of AP [1]. Scholars have found that the main pathogenesis of AP is the undesired overactivation of trypsinogen in pancreatic cells [5]. However, the mechanisms regulating AP progression remain a matter of clarification.

Exosomes are vesicles secreted by cells that have a double plasma membrane structure, which carries specific cytokines of mother cells, including mRNA, miRNA, and lncRNA [6]. The role of exosomes in pancreatitis has been explored. For example, exosomal lnc-MMP2-2 increases vascular permeability and promotes lung cancer progression by promoting MMP2 expression [7]. Lnc-MKRN2-42 : 1 in exosomes from plasma samples is positively correlated with MDS-UPDRS III scores in patients with Parkinson's disease, and it may be involved in the development of Parkinson's disease [8]. Only one paper has reported the involvement of exosomal lncRNA in the progression of acute pancreatitis, that is, rhodopsin suppresses acute pancreatitis by regulating the expression of cellular and exosomal lncRNA TUG1 [9]. The effect of lncRNA in NAFLD-derived exosomes on pancreatitis has not been explored previously.

Long noncoding RNA (lncRNA) is a special RNA molecule with a transcript length of more than 200 nucleotides and no protein-coding function [10]. The metastasis-associated lung adenocarcinoma transcript 1 (MALAT1), also is a long noncoding RNA [11]. One prior study found that lncRNA MALAT1 in exosomes from conditioned medium facilitates ischemic wound healing [12]. According to research, MALAT1 plays an important role in pancreatitis. Extracellular vesicle-shuttled MALAT1 promotes macrophage M1 polarization through miR-181a-5p/HMGB1 to induce acute pancreatitis [13]. MATAL1/miR-194/YAP1 has a regulatory effect on the progression of AP [14]. However, no data have been presented to verify the effect of NAFLD-derived lncRNA MALAT1 on the regulation of AP. It is reported that lncRNAs are involved in the progression of acute pancreatitis [15, 16], but the influence of NAFLD-derived MALAT1 in acute pancreatitis remains blurry.

In this study, the research aimed to uncover the influence of lncRNA MALAT1 in AP, and we hypothesized that NAFLD-derived MALAT1 could potentially affect the progression of AP and conduct a series of experiments to explore whether NAFLD-derived MALAT1 affects the progression of AP. The study is intended to provide a theoretical basis and potential targets for the treatment of clinical AP patient.

## 2. Materials and Methods

### 2.1. Isolation and Characterization of Exosomes

In this experiment, we borrowed the method of Thery *et al.* [17] to isolate exosomes. ExoQuick-TC (System Biosciences, Mountain View, CA) was used for the isolation of exosomes. We identified the isolated exosomes by transmission electron microscopy, western blot analysis, and nanoparticle tracking analysis.

### 2.2. Cell Culture

HepG2 and AR42J were obtained from the American Type Culture Collection (ATCC, Manassas, US). The cell lines HepG2 were cultured in Dulbecco's Modified Eagle Medium (DMEM) (Gibco, Paisley, UK, US) medium containing 10% fetal bovine serum (FBS, HyClone, UT, USA) for 24 h. AR42J were cultured in F–12K (Gibco) medium containing 20% FBS (HyClone) for 24 h. Then, the cells were incubated in an incubator at 37°C with 5% CO_2_.

### 2.3. Cell Transfection

The sequences of si-NC and si-MALAT1 were obtained by GenePharma (Shanghai, China). HepG2 cells were transfected with si-NC and si-MALAT1 using Lipofectamine 2000 (Invitrogen, CA, USA) for 24 h. The transfected cells were used for further study.

### 2.4. Establishment of the NAFLD Cell Model and AP Cell Model

HepG2 treated with or without 1 mM free fatty acid (FFA, containing 2 : 1 v/v oleic acid and palmitic acid) for 24 h was used for subsequent experiments. In addition, AR42J cells cultured for 24 h were incubated with 20 nM caerulein (#C9026, Sigma-Aldrich, St Louis, MO, USA) for 48 h for the construction of AP cell model.

### 2.5. Oil Red O Staining

After fixing HepG2 cells in 10% formalin for 5 min, they were incubated with Oil Red O reagent for 30 min. The stained cells were then counterstained with hematoxylin for 1 min, and sections were dewaxed and rehydrated in xylene. Tissue sections were then incubated in Oil Red O reagent for 30 minutes and counterstained with hematoxylin for 1 min. Sections were finally imaged on a fluorescence microscope (IX-51, Olympus, Tokyo, Japan).

### 2.6. Quantitative Real-Time Reverse Transcription-Polymerase Chain Reaction (qRT-PCR)

For the examination of the MALAT1 expressions, isolated from exosomes by TRIzol reagent (Ambion, Austin, TX). 1 *μ*g of total RNA was reverse transcribed using the all-in-one miRNA qRT-PCR detection kit (GeneCopoeia Rockville, MD, USA). The qRT-PCR was performed on the CFX96 PCR detection system (Bio-Rad Laboratories, Hercules, CA, USA). The sequences used in qRT-PCR were presented as follows: MALAT1: 5′-GCT CTG TGG TGT GGG ATT GA-3' (F) and 5′-GTG GCA AAA TGG CGG ACT TT-3' (*R*); GAPDH: 5′-CCA GGT GGT CTC CTC TGA-3' (F) and 5′-GCT GTA GCC AAA TCG TTG T-3′(R). The 2-^ΔΔ^Ct method was adopted to analyze relative fold change [18].

### 2.7. Western Blot

Cells were completely lysed in lysis buffer (Takara, Shiga, Japan) and extracted nuclear proteins and cytoplasmic proteins. The BCA protein assay kit (Pierce, Rockford, IL) was used to detect the corresponding protein densities. 50 *μ*g of the sample was taken for SDS-PAGE electrophoresis and transferred to the PVDF membrane. Then, membranes were blocked with 5% skim milk. Membranes were then incubated with the corresponding primary antibodies, including anti-CD9 antibody (ab178860, 1 : 1000, Abcam, Cambridge, MA, USA), anti-CD63 antibody (ab188570, 1 : 5000, Abcam), anti- CD81 antibody (ab3778; 1 : 200，Abcam), anti-CYP2E1 antibody (ab52915, 1 : 10000, Abcam), anti-YAP-13 antibody (ab51072, 1 : 1000, Abcam), anti-phosphorylated-YAP antibody (ab185722, 1 : 1000, Abcam), anti-LC3II antibody (ab41037, 1 : 250, Abcam), anti-LC3I antibody (ab32360, 1 : 5000, Abcam), anti-LATS1 antibody (ab32452, 1 : 2000, Abcam), and anti-*β*-actin antibody (ab8226, 1 : 10000, Abcam) overnight at 4°C. *β*-actin was used as internal controls. Then, membranes were incubated with horseradish peroxidase-labeled secondary antibody (ab6721, 1 : 2000, Abcam) for 1 h at room temperature. Then, the specific protein bands were visualized using an enhanced chemiluminescent (ECL; Millipore, Shanghai, China).

### 2.8. Enzyme-Linked Immunosorbent Assay (ELISA)

TNF-*α* ELISA and IL-6 ELISA kits (Thermo, MA, USA) were performed to measure TNF-*α* and IL-6 secretion and finally the specific levels of TNF-*α* and IL-6 were determined by a standard curve.

### 2.9. Statistical Analysis

Data from at least three independent experiments were exhibited as mean ± SD, analyzed by SPSS 17.0 statistical software. Paired Student's t-test was performed to compare the differences between the two groups. One-way ANOVA along with Bonferroni's posttest was used to analyze the differences between more than two groups. *P* value < 0.05 was considered statistically significant.

## 3. Results

### 3.1. MALAT1 Is Upregulated in NAFLD-Derived Exosomes

To assess whether the NAFLD cell model was successfully constructed, we examined the lipid deposition and triglyceride content in the hepatocytes and in the culture medium supernatant, respectively. The results indicated lipid deposition was remarkably increased in the FFA group (Figure 1(a)). The TG content was significantly elevated in the supernatant of HepG2 cell medium compared with the Control group (Figure 1(b), *p* < 0.001). Extracellular vesicles isolated from cell supernatant were characterized by the TEM. Vesicular morphology and a diameter between 50 and 150 nm were evident in TEM images (Figure 1(c)). Besides, we found that the isolated exosomes from the Control group and the FFA group expressed not only the exosomal markers CD9, CD63, and CD81 as expected but also hepatocyte marker proteins CYP2E1 (Figure 1(d)). We also examined the expression of MALAT1 in exosomes and found that the expression of MALAT1 was significantly increased after FFA induction, in contrast to in exosomes produced from HepG2 cells without FFA induction (Figure 1(e), *p* < 0.001). We cocultured the exosomes with pancreatic cells AR42J and measured the secretion levels of inflammatory factors in the pancreatic cell medium. The results showed the levels of IL-6 and TNF-*α* in the FFA group were obviously higher (Figure 1(e), *p* < 0.001). These results suggest that these hepatocytes are their primary source of the isolated exosomes wrapped in MALAT1. All illustrated that MALAT1 is upregulated in NAFLD-derived exosomes.

### 3.2. NAFLD-Derived Exosomes Exacerbate the Inflammatory Response and Inhibit YAP Phosphorylation and Autophagy in Pancreatic Cells

To investigate whether NAFLD-derived exosomes regulate the inflammatory response, YAP expression, and autophagy in pancreatic cells, we then cocultured exosomes with AR42J pancreatic cells.  Figure 2(a) reveals inflammatory factors IL-6 and TNF-*α* level were increased in pancreatic cell cultures cocultured with exosomes relative to controls (*p* < 0.001). The level of YAP/p-YAP was obviously increased in the FFA group when compared with the Control group (Figure 2(b), *p* < 0.001). The levels of LC3II/LC3I in pancreatic cells were largely decreased after coculture of pancreatic cells and exosomes (Figure 2(c), *p* < 0.001). All of the above illustrates that NAFLD-derived exosomes promote the inflammatory response and inhibit YAP phosphorylation and autophagy in pancreatic cells.

### 3.3. NAFLD-Derived Exosomes Inhibit Hippo-YAP Pathway, Suppress Autophagy, and Promote Inflammatory Responses in Pancreatic Cells via MALAT1

Based on the upregulation of MALAT1 in NAFLD-derived exosomes, the effects of NAFLD-derived exosomes on the inflammatory response and autophagy of pancreatic cells were investigated, as well as we speculated that MALAT1 may be involved in the regulatory process of exosomes in pancreatic cells.  Figure 3(a) shows that the successful knockdown of MALAT1 in HepG2 cells (*p* < 0.001). Meanwhile, the MALAT1 level was significantly reduced in the exosomes extracted from FFA-induced HepG2 cells transfected with si-MALAT1 in relative to the FFA group (Figure 3(b), *p* < 0.001). Moreover, MALAT1 expression was elevated in pancreatic cells after cocultured with FFA-induced exosomes, and silencing MALAT1 reversed the increase in MALAT1 levels induced by FFA induction (Figure 3(c), *p* < 0.001). We further explored the effects of silencing MALAT1 on Hippo-YAP pathway, autophagy, and inflammation in pancreatic cells. Figures 3(d) and 3(e) show that LATS1 was much lower in the FFA group than that in the Control group (*p* < 0.001), while silencing MALAT1 effectively recovered this status (*p* < 0.001); the level of YAP/p-YAP showed an opposite trend (*p* < 0.01, *p* < 0.001). As shown in Figures 3(f) and 3(g), the levels of the LC3II/LC3I were reduced in the FFA group (*p* < 0.001), which was partly restored in the FFA + si-MALAT1 group (*p* < 0.01). Besides, FFA induction resulted in increased levels of IL-6 and TNF-*α* (*p* < 0.001), and silencing MALAT1 followed by FFA induction reversed the augment in IL-6 and TNF-*α* levels induced by FFA induction (Figure 3(h), *p* < 0.01). These suggested that NAFLD-derived exosomes inhibit the Hippo-YAP pathway, suppress autophagy, and promote inflammatory responses in pancreatic cells via upregulating MALAT1.

### 3.4. MALAT1 Exacerbates AP via Inhibiting Autophagy by Upregulating YAP

To further confirm the underlying molecular mechanism of MALAT1 in regulating AP, we then examined the effects of MALAT1 on YAP and autophagy in an *in vitro* model of AP. The results first showed the increased MALAT1 in pancreatic cells transfected with MALAT1 and the decreased MALAT1 in pancreatic cells transfected with si-MALAT1, indicating the successful overexpression and knockdown of MALAT1 in the *in vitro* model of AP (Figures 4(a) and 4(b), *p* < 0.001). Clearly, the *in vitro* model of AP with MALAT1 overexpression showed the increased expression of IL-6 and TNF-*α* levels (*p* < 0.01), while silencing MALAT1 decreased the IL-6 and TNF-*α* levels (Figure 4(c), *p* < 0.05). Besides, the level of LC3II/LC3I was reduced in the AP cell model with MALAT1 overexpression (*p* < 0.001), but such trend was significantly restored by the YAP inhibitor CA3 (Figures 4(d) and 4(e), *p* < 0.01). The inhibition of YAP CA3 inhibited the increase of IL-6 and TNF-*α* level caused by MALAT1 (Figure 4(f), *p* < 0.01). The above indicated that MALAT1 exacerbates AP via inhibiting autophagy by promoting YAP.

## 4. Discussion

Exosomes perform cell-to-cell actions by delivering exosomal contents and regulating receptor cell [19–21]. Almost all types of cells can secrete exosomes, and exosomes are also widely present in body fluids [19, 22, 23]. The *κ* stem cell-derived exosomes prevent cardiac insufficiency via lncRNA MALAT1/NF-*κ*B/TNF [24]. Exosomal Hic-5 regulates osteosarcoma phenotype [25]. Human mesenchymal stem cells promote ischemic repairment and angiogenesis of diabetic foot through exosomal miRNA-21-5p [26]. In NAFLD, stressed/damaged hepatocytes release large amounts of EVs, leading to the development of inflammation, fibrogenesis, and angiogenesis, which are key pathobiological processes in the progression of liver disease [27]. In this paper, we demonstrated that the FFA-induced NAFLD cell model secretes a large number of exosomes, when cocultured with AR42J pancreatic cancer cells, and inhibits YAP phosphorylation and autophagy in AR42J.

MALAT1 is the first lncRNA found to be involved in the occurrence and development of various cancers. MALAT1 can induce the metastasis and invasion of various cancer cells [28, 29]. Studies report that MALAT1 has pro-inflammatory effects, which was able to aggravate cardiac inflammation [30] and promote EC inflammation [31]. Furthermore, exosomal MALAT1 derived from HUVECs promoted inflammatory response in atherosclerotic mice [32]. Herein, we found that MALAT1 was upregulated in NAFLD-derived exosomes. Coculture of exosomes with AR42J pancreatic cells increased inflammatory factor levels in AR42J cell culture medium. Our subsequent study confirmed that NAFLD hepatocyte-derived exosomes promoted inflammatory responses in pancreatic cells through MALAT1. Our findings are consistent with those reported in previous studies that MALAT1 has pro-inflammatory effects.

The Hippo signaling pathway is a key regulator in the pathway, which consists of a series of conserved kinases that control organ size primarily by regulating cell proliferation and apoptosis [33], which have been researched in pancreas development and pancreatic cancer [34, 35]. Moreover, the activation of Hippo signaling pathway participated in regulating ferroptosis in acute lung injury [36]. However, the function of Hippo signaling pathway in AP is still unclear. YAP (Yes-associated protein) is a major downstream effector of the Hippo pathway and mediates the effects of the Hippo pathway by regulating the gene expression [37, 38]. The Hippo-YAP axis has been reported to have a nonnegligible role in regulating autophagy [39]. It is well known that Hippo plays an important role in the occurrence of inflammation. Naringin protects endothelial cells from apoptosis and inflammation by regulating the Hippo-YAP pathway [40]. Hippo/YAP pathway plays a critical role in effect of GDNF against A*β*-induced inflammation in microglial cells [41]. The inhibition of Hippo/YAP signaling pathway is required for magnesium isoglycyrrhizinate to ameliorate hepatic stellate cell inflammation and activation [42]. Our study shows that NAFLD hepatocyte-derived exosomes inhibit Hippo-YAP pathway and autophagy in pancreatic cells via MALAT1. The regulatory effect of MALAT1 on the Hippo-YAP pathway has been reported in the literature. Downregulation of MALAT1 inhibits the development of pancreatic cancer by activating the Hippo-YAP pathway [43]. MALAT1 interference decreased collagen accumulation and inflammation in high-glucose CFs and DCM mice [44]. Downregulation of MALAT1 suppressed the proliferation and adhesion of myeloma cells [45]. Furthermore, MALAT1 has been found to have regulatory effects on autophagy in a range of diseases. MALAT1 enhances the apoptosis of cardiomyocytes [46]. Long noncoding RNA MALAT1 affects the development of endometriosis [47] and promoted cell proliferation, yet inhibited apoptosis in colorectal cancer cells [48]. The results of this experiment are consistent with the theory and consistent with the existing literature reports.

We subsequently confirmed through rescue experiments that MALAT1 exacerbates AP by promoting YAP and thereby inhibiting autophagy. The involvement of MALAT1 in the progression of pancreatitis has been documented. An important research study demonstrated that MALAT1/miR-181a-5p/HMGB1 induced AP [13]. Baicalin can affect the expression of miR-15a to prevent the occurrence of AP. Long noncoding RNA MALAT1, regulated by baicalin, targets miR-15a [49]. MALAT1 affects pancreatic cancer progress [50] and acts on AP via miR-194/YAP1 [14]. Treatment of MALAT1 overexpressing pancreatic cancer cells with CA3 in our research revealed that inhibition of YAP reversed the inhibition of autophagy and promotion of inflammatory response induced by MALAT1 overexpression. The role of Hippo pathway has been studied in the pancreas. Hippo signaling not only regulates pancreatic development by inactivating YAP [51], but also affects the differentiation and maintenance of the exocrine pancreas [52]. Proliferative and antiapoptotic action of exogenously introduced YAP in pancreatic cells [53]. YAP levels have a clear upward trend in alveolar and ductal cells of mice with pancreatitis and may be involved in regulating pancreatic tissue regeneration and stellate cell function [54]. Our study found that NAFLD-derived MALAT1 inhibits autophagy to further promote inflammatory responses by suppressing the Hippo-YAP pathway in pancreatic cells.

## 5. Conclusion

Taken together, our research is the first to clarify that exosomal lncRNA MALAT1 originating from NAFLD exacerbated pancreatic cell inflammation by regulating YAP inhibition of autophagy. This molecule may bring a major breakthrough in the clinical treatment of NAFLD. However, some potential mechanisms and Hippo signaling pathway regulation in AP are worthy further investigated.

## Figures and Tables

**Figure 1:** Increased expression of MALAT1 in NAFLD-derived exosomes exacerbates the inflammatory response in pancreatic cells. (a) Lipid deposition in NAFLD cell models was detected using Oil Red O staining. (b) TG in the supernatant of NAFLD cell model culture medium was detected by the ELISA assay. (c) Collected exosomes were observed by transmission electron microscopy. (d) CD9, CD63, and CD81 protein levels and liver marker CYP2E1 were investigated by western blot. (e) Expression of MALAT1 in exosomes was probed by qRT-PCR. ^*∗∗∗*^*p* < 0.001 vs. Control group. TG: triglycerides.

**Figure 2:** NAFLD-derived exosomes from nonalcoholic fatty liver activate YAP and inhibit autophagy in pancreatic cells. (a) The ELISA assay was used to detect levels of IL-6 and TNF-*α*. (b) The protein expression of YAP and phosphorylated YAP were detected by western blot. (c) The protein expression of LC3II and LC3I was detected by western blot. ^*∗∗∗*^*p* < 0.001 vs. Control group.

**Figure 3:** NAFLD-derived exosomes activate the Hippo-YAP pathway, suppress autophagy and inflammatory responses in pancreatic cells via MALAT1. (a) qRT-PCR was used to analyze MALAT1 levels in Human hepatocytes HepG2 following si-NC and si-MALAT1 transfection. (b) qRT-PCR was used to analyze MALAT1 levels in exosomes. (c) qRT-PCR analysis of MALAT1 expression in AR42J pancreatic cells after co-culture with NAFLD-derived exosomes. (d, e) Hippo-YAP pathway-associated protein LATS1, YAP and phosphorylated YAP were detected using western blot assay. (f, g) Autophagy-associated proteins LC3II and LC3I were measured by western blot assay. (h) ELISA assay was performed on the secretion levels of IL-6 and TNF-*α*. ^*∗∗∗*^*p* < 0.001 vs. si-NC group/NC group/Control group; ^##^*p* < 0.01 and ^###^*p* < 0.001 vs. FFA group.

**Figure 4:** MALAT1 further inhibits autophagy by promoting YAP and eventually exacerbates AP. (a, b) The relative expression of MALAT1 in AR42J pancreatic cells transfected with MALAT1 and si-MALAT1 were examined using qRT-PCR assay. ^*∗∗∗*^*p* < 0.001 vs. NC/si-NC group. (c) Levels of IL-6 and TNF-*α* was detected by ELISA assay in AR42J pancreatic cells treated with caerulein and/or transfected with MALAT1 and si-MALAT1. ^*∗*^*p* < 0.05 and ^*∗∗∗*^*p* < 0.001 vs. NC group; ^##^*p* < 0.01 vs. Caerulein group. (d, e) The relative protein expression of LC3II and LC3I was measured by the western blot assay. (f) The levels of IL-6 and TNF-*α* were determined utilizing ELISA assay. ^*∗∗∗*^*p* < 0.01 vs. NC group; ^##^*p* < 0.01 vs. MALAT1 group.

## Data Availability

The datasets used and analyzed during the current study are available from the corresponding author upon reasonable request.
